The article "Chinese Herbal Medicine as an Adjunctive Therapy Improves the Survival Rate of Patients with Ischemic Heart Disease: A Nationwide Population-Based Cohort Study" was published in 2022. Journal: Evid Based Complement Alternat Med.

# Chinese Herbal Medicine as an Adjunctive Therapy Improves the Survival Rate of Patients with Ischemic Heart Disease: A Nationwide Population-Based Cohort Study

**DOI:** 10.1155/2022/5596829

**Published:** 2022-07-04

**Authors:** I.-Ling Hung, Chia-Jung Chung, Wen-Long Hu, Yen-Nung Liao, Chung-Y. Hsu, Jen-Huai Chiang, Yu-Chiang Hung

**Affiliations:** ^1^Department of Chinese Medicine, Kaohsiung Chang Gung Memorial Hospital and Chang Gung University College of Medicine, Kaohsiung, Taiwan; ^2^Department of Chinese Medicine, Jen-Ai Hosiptal, Taichung, Taiwan; ^3^Kaohsiung Medical University College of Medicine, Kaohsiung, Taiwan; ^4^Fooyin University College of Nursing, Kaohsiung, Taiwan; ^5^Graduate Institute of Biomedical Sciences, China Medical University, Taichung, Taiwan; ^6^Management Office for Health Data, China Medical University Hospital, Taichung, Taiwan; ^7^College of Medicine, China Medical University, Taichung, Taiwan

## Abstract

**Background:**

Ischemic heart disease (IHD) related to cardiovascular or cerebrovascular disease is the leading cause of mortality and an important issue of public health worldwide. The cost of long-term healthcare for IHD patients may result in a huge financial burden.

**Objectives:**

To analyze the medical expenditure incurred for and survival of IHD patients treated with Chinese herbal medicine (CHM) and Western medicine.

**Methods:**

Subjects were randomly selected from the National Health Insurance Research Database in Taiwan. The Cox proportional hazards regression model, Kaplan–Meier estimator, logrank test, chi-square test, and analysis of variance were applied. Landmark analysis was used to assess the cumulative incidence of death in IHD patients.

**Results:**

We identified 11,527 users of CHM combined with Western medicine and 11,527 non-CHM users. CHM users incurred a higher medical expenditure for outpatient care within 1 (24,529 NTD versus 18,464 NTD, *P* value <0.0001) and 5 years (95,345 NTD versus 60,367 NTD, *P* value <0.0001). However, CHM users had shorter hospitalizations and lower inpatient medical expenditure (7 days/43,394 NTD in 1 year; 11 days/83,141 NTD in 5 years) than non-CHM users (11 days/72,939 NTD in 1 year; 14 days/107,436 NTD in 5 years). The CHM group's adjusted hazard ratio for mortality was 0.41 lower than that of the non-CHM group by Cox proportional hazard models with time-dependent exposure covariates. Danshen, Huang qi, Niu xi, Da huang, and Fu zi were the most commonly prescribed Chinese single herbs; Zhi-Gan-Cao-Tang, Xue-Fu-Zhu-Yu-Tang, Tian-Wang-Bu-Xin-Dan, Sheng-Mai-San, and Yang-Xin-Tang were the five most frequently prescribed herbal formulas in Taiwan.

The article "Chinese Herbal Medicine as an Adjunctive Therapy Improves the Survival Rate of Patients with Ischemic Heart Disease: A Nationwide Population-Based Cohort Study" was published in 2022. Journal: Evid Based Complement Alternat Med.

**Conclusions:**

Combining Chinese and Western medicine can reduce hospital expenditure and improve survival for IHD patients.

## 1. Introduction

Ischemic heart disease (IHD) is a major cause of myocardial infarction (MI) and ischemic stroke, which are the main causes of death and disability in the world [1, 2]. IHD has become the world's most important issue of public health and the largest cause of death due to noncommunicable disease, accounting for more than 50%. The World Health Organization (WHO) estimates that 17.6 million people died of IHD worldwide in 2012 [3]. In the 2000s, the mortality rates associated with IHD were 50% and 25% in developed and developing countries, respectively. Approximately 25 million people will be diagnosed with IHD in 2020, and the condition is expected to be the main cause of death worldwide (about 30%) [4, 5].

Although the mortality rates associated with IHD have declined due to risk-factor modification (decreased exposure to tobacco smoke and improvement of hypertension, dyslipidemia, and diabetes control) and timely treatment with thrombolysis and primary angioplasty for acute IHD events in recent decades [2], it still is the leading cause of death in Taiwan. Furthermore, as IHD is the most common underlying cause of heart failure, the cost of long-term healthcare for IHD patients may result in a huge financial burden. In patients with a history of MI, the rate of cardiovascular mortality in the absence of treatment is about 5% per year after the first MI and 10% per year after a subsequent MI; this increase may persist for the rest of a patient's life [6]. According to 2016 mortality data from the National Center for Health Statistics, there were 363,452 deaths in Taiwan due to IHD and 111,777 deaths due to MI [7]. Although the annual death rate attributable to IHD has declined by 31.8% and the actual number of deaths declined by 14.6% from 2006 to 2016, IHD remains the primary cause of death worldwide [7].

Many patients seek natural remedies for IHD, and traditional Chinese medicine (TCM) is a common choice for treatment. The origin of TCM can be traced back thousands of years in China and other areas of East Asia. From the perspective of TCM, the pathogeneses of IHD are blood stasis and/or phlegm retention, and IHD may result in qi deficiency and inadequacy of Yin and Yang. It has been reported that some Chinese herbs may improve blood perfusion and protect against oxidative stress associated with IHD [8]. However, clinical evidence regarding the efficacy of TCM for the treatment of IHD is limited.

Taiwan is unique in that TCM has been universally covered under the National Health Insurance (NHI) program since its establishment in 1995. The program covers 99.6% of 23.16 million people enrolled in 2011. Chinese herbal medicine (CHM) is part of an integrated system of primary healthcare known as TCM, which is covered by the NHI program. The aim of the present study was to analyze the expenditure and survival of IHD patients treated with CHM and determine the prescription patterns of CHM for IHD.

The article "Chinese Herbal Medicine as an Adjunctive Therapy Improves the Survival Rate of Patients with Ischemic Heart Disease: A Nationwide Population-Based Cohort Study" was published in 2022. Journal: Evid Based Complement Alternat Med.

## 2. Materials and Methods

### 2.1. Data Source

In 1995, Taiwan's compulsory universal NHI program was developed by the National Health Insurance Administration. The NHI program covers 99.6% of the Taiwanese population and insures not only Western medicine prescriptions but also TCM services, including herbal medicine, acupuncture, and moxibustion. In this study, we used data from the Longitudinal Health Insurance Database, which includes the health claim data of 1 million individuals registered with the NHI program. The database contains all longitudinal reimbursement information, as well as gender, birth date, medications, and diagnosis codes based on the International Classification of Diseases, Ninth Revision, Clinical Modification (ICD-9-CM). This study was designed as a population-based study of a sample of 1 million subjects selected at random from the 22 million beneficiaries of the NHI program in Taiwan. The study design was approved by the Institutional Review Board of China Medical University (CMUH104-REC2-115).

### 2.2. Study Population

Patients newly diagnosed by a cardiologist with IHD between 2000 and 2010 were identified as the IHD cohort. These IHD patients had at least two ambulatory or inpatient claims with a diagnosis of ICD-9-CM code 411-414 during this period. Cardiologists would identify new IHD cases through asking about patient's symptoms, taking patient's medical history, reviewing patient's risk factors, performing a physical exam, and checking some tests as electrocardiograph, echocardiogram, or computed tomography scan. Study subjects with the diagnosis of IHD from 1996–1999 were excluded at the baseline to begin the identification of patients with IHD newly diagnosed from 2000–2010. Therefore, most prevalence cases of IHD were not likely included in the study cohort. We excluded patients younger than 20 years of age and those who had withdrawn from the NIH program within a year of follow-up. The IHD patients who had accepted Western medicine treatment with at least one CHM outpatient clinical record during the follow-up period were defined as CHM users, whereas those who had only accepted Western medicine with no CHM outpatient records after the initial IHD diagnosis date were defined as non-CHM users (Figure 1). The index date was defined as the initial IHD diagnosis date [9–11]. The wash-out period was about 1 year. Because the initial status of patients with incident IHD may be a confounding factor to the outcome, 1 : 1 propensity score matching was applied to eliminate baseline differences between CHM and non-CHM users when IHD was diagnosed, including sex, age (per 5 years), index year, and initial IHD diagnosis year. Both cohort groups had the same distributions of sex and age.

The article "Chinese Herbal Medicine as an Adjunctive Therapy Improves the Survival Rate of Patients with Ischemic Heart Disease: A Nationwide Population-Based Cohort Study" was published in 2022. Journal: Evid Based Complement Alternat Med.

### 2.3. Assessment

The primary outcome of this study was IHD-related death and hospitalization. The covariate assessment, including age, sex, and comorbidities, was also considered. Sociodemographic factors included age and sex. Age was divided into three groups: 20–39 years, 40–64 years, and ≧65 years. Baseline comorbidities were considered present if ICD-9-CM codes were included in at least two ambulatory claims or one inpatient claim before the initial diagnosis of IHD, including hyperlipidemia (ICD-9-CM code 272), hypertension (ICD-9-CM code 401), diabetes mellitus (ICD-9-CM code 250), and stoke (ICD-9-CM code 433-438). Charlson's comorbidity index score (CCI) was also calculated as summaries of IHD-related comorbidities (shown at the bottom of Table 1).

### 2.4. Variables for Expenditures and Visits

The database contained information regarding the dates of visits, the medical facility visited, the department visited, the type of copayment, and the amounts billed and paid. All visits within 1 and 5 years, particularly after the index date, were analyzed for the expenditures of outpatient and inpatient visits with ICD-9-CM code 411-414.

### 2.5. Statistical Analysis

Differences in demographic characteristics and comorbidities between the study and comparison cohorts were examined using the chi-squared test for categorical variables and analysis of variance (ANOVA) or two-sample *t*-tests for continuous variables. We performed 1 : 1 propensity score matching between CHM users and non-CHM users, including sex, age (per 5 years), index year, and initial IHD diagnosis year. The means of outpatient and inpatient visits and medical expenditure for CHM users and non-CHM users were compared using the Wilcoxon rank-sum test. Univariate and multivariate time-dependent Cox proportional hazards models were used to evaluate mortality hazard ratios (HRs) for CHM users. We estimated HRs and their 95% confidence intervals (CIs) by adjusting for age, gender, hyperlipidemia, diabetes mellitus, and stroke in a Cox proportional hazards model. The Kaplan–Meier estimator and logrank test were applied to compare the survival distributions of IHD patients in both groups. A 5-year landmark analysis was used to assess the cumulative incidence of death in IHD patients. Statistical analysis was performed, and figures were created using SAS 9.4 (SAS Institute, Cary, NC) software. *P* < 0.05 in two-tailed tests indicated statistical significance.

The article "Chinese Herbal Medicine as an Adjunctive Therapy Improves the Survival Rate of Patients with Ischemic Heart Disease: A Nationwide Population-Based Cohort Study" was published in 2022. Journal: Evid Based Complement Alternat Med.

## 3. Results

Table 1 shows the baseline characteristics of IHD patients in the CHM-user and non-CHM-user groups. Using data from January 2000 to December 2010, we identified 20,192 CHM users and 20,192 non-CHM users. The mean ages were 63.4 ± 13.1 years and 63.5 ± 13.2 years for CHM users and non-CHM users, respectively. The median mean follow-up periods were 8.12 and 6.00 years for the CHM-user group and non-CHM-user group, respectively. The mortality rate for the CHM-user group was significantly lower than for the non-CHM-user group.

Table 2 shows the clinical visits of outpatients and inpatients in the two groups for the first 1 and 5 years. CHM users had significantly more outpatient visits than non-CHM users within 1 and 5 years (1 year: 29 visits versus 24 visits, *P* value <0.0001; 5 years: 133 visits versus 94 visits, *P* value <0.0001). CHM users also had higher medical expenditure for outpatient care within 5 years (123,496 NTD versus 60,367 NTD, *P* value <0.0001) after incident IHD. However, CHM users had fewer hospitalization days (6 days in 1 year and 11 days in 5 years) and lower medical expenditure (67,098 NTD versus 105,608 NTD) in 1 year than non-CHM users.

To identify prescription patterns, we further analyzed the Chinese herbal formulas prescribed by TCM doctors to treat patients with IHD (Table 3). The five most frequently prescribed herbs were Danshen (678 times in frequency and 7,730 person-days of administration), Huang qi (264 times and 2,610 person-days), Niu xi (144 times and 2,483 person-days), Da huang (137 times and 1,435 person-days), and Fu zi (137 times and 1,302 person-days). Zhi-Gan-Cao-Tang (459 times in frequency and 4,861 person-days), Xue-Fu-Zhu-Yu-Tang (338 times and 3,332 person-days), Tian-Wang-Bu-Xin-Dan (202 times and 2,546 person-days), Sheng-Mai-San (178 times and 2,404 person-days), and Yang-Xin-Tang (137 times and 955 person-days) were the five most frequently prescribed herbal formulas.

Table 4 shows the HRs of the ten most frequently prescribed CHM single herbs and formulas. We also estimated the HRs of mortality for CHM users and non-CHM users using the Cox proportional hazards model. After adjusting for age, sex, hyperlipidemia, diabetes mellitus, and stroke, the HR of mortality in the CHM group was 0.45 (95% CI: 0.42–0.48), 55% lower than that in the non-CHM group. Adjusted HRs of mortality in the CHM user compared with those in the non-CHM user by Cox proportional hazard models with time-dependent exposure covariates are 0.08 (95% CI: 0.06–0.11) in Table 5. Compared with the non-CHM group, there was a significantly lower risk of mortality for those using Danshen (HR: 0.28, 95% CI: 0.14–0.56), Xue-Fu-Zhu-Yu-Tang (XFZYT) (HR: 0.23, 95% CI: 0.09–0.62), Zhi-Gan-Cao-Tang (ZGCT) (0.51, 95% CI: 0.62–0.98), and Tian-Wang-Bu-Xin-Dan (TWBXD) (HR: 0.29, 95% CI: 0.09–0.90). IHD patients with CHM treatment had a lower incidence rate and hazard ratio of mortality than IHD patients without CHM treatment stratification by gender, age, baseline comorbidity, and Charlson comorbidity index in Table 6.

The article "Chinese Herbal Medicine as an Adjunctive Therapy Improves the Survival Rate of Patients with Ischemic Heart Disease: A Nationwide Population-Based Cohort Study" was published in 2022. Journal: Evid Based Complement Alternat Med.

The longer survival time of the CHM group is shown in the Kaplan–Meier plots in Figure 2. The logrank test and Kaplan–Meier curve of the 10-year survival rate revealed a statistically significant difference between CHM users (survival rate 91%) and non-CHM users (survival rate 82%). A landmark analysis revealed that the cumulative incidence of death in the early period (0–5 years) was significantly higher in non-CHM users than in CHM users. However, Figure 3(a) had no these findings in the late period (5–12 years).  Figure 3(b) revealed the adjusted HR of CHM during different follow-up periods in the landmark analysis.

## 4. Discussion

IHD patients within the CHM group had lower mortality, fewer days of hospitalization, and lower inpatient medical expenditure during the 1- and 5-year follow-ups compared with the non-CHM group. IHD patients in the CHM group had longer survival times than those in the non-CHM group. These findings indicate that the integration of CHM and Western medicine may yield an appropriate treatment for IHD patients. Chinese herbs and formulas may be used as a complementary therapy for the treatment of patients with IHD.

CHM users had significantly more outpatient visits and medical expenditure than non-CHM users within 1 and 5 years. When IHD patients see Western medicine doctors and Chinese medicine physicians, taking both traditional drugs and Chinese herbs, the medical expenses will be greater than the cost of treatment with only Western medicine. However, after receiving integrated CHM and Western medicine treatments at the outpatient clinic, the IHD patients' illnesses were relieved; they were hospitalized for a shorter period and had a lower risk of mortality. Integrating CHM and Western medicine treatments may reduce hospitalization and death of IHD patients at least within 1 year.

Not only CHM formulas but also single herbs prescribed by TCM physicians significantly decreased the HRs related to mortality risk in patients with IHD. It must be noted that TCM treatment is based on TCM syndrome differentiation and may vary with the experience of TCM physicians. According to TCM theory, IHD is caused by blood stasis and/or phlegm retention, and it may result in qi deficiency and inadequacy of Yin and Yang. Danshen, San qi, Hong hua, and Xue-Fu-Zhu-Yu-Tang (XFZYT) activate blood circulation and are often used for the treatment of blood-stasis syndrome. Huang qi, ZGCT, Tian-Wang-Bu-Xin-Dan (TWBXD), Sheng-Mai-San (SMS), and Yang-Xin-Tang (YXT) benefit qi, activate heart-yang, and nourish heart-yin. Based on our findings, the use of the most frequent single herb (Danshen) and CHM formula (ZGCT, XFZYT, and TWBXD) is associated with a decrease in mortality risk.

The article "Chinese Herbal Medicine as an Adjunctive Therapy Improves the Survival Rate of Patients with Ischemic Heart Disease: A Nationwide Population-Based Cohort Study" was published in 2022. Journal: Evid Based Complement Alternat Med.

Danshen, also known as *Salvia miltiorrhiza*, has been widely used in Asian countries to treat a diverse range of cardiovascular diseases, including angina pectoris and MI [12, 13]. Danshensu (DSS), one of the soluble agents extracted from Danshen, has been reported to protect the heart against ischemic/reperfusion injury by reducing reactive oxygen species generation and inhibiting apoptosis [12, 14]. Fan et al. [15] demonstrated that the cardioprotective effects of DSS were mediated by activation of the mammalian target of rapamycin signaling pathway. Salvianolic acid B, another major soluble agent derived from Danshen, may reduce infarction size by boosting autophagy and neovascularization to stave off apoptosis [16]. Tanshinone IIA (Tan IIA), a derivative of phenanthrenequinone isolated from Danshen, elicited signiﬁcant cardioprotective eﬀects by promoting angiogenesis in an MI rat model. Tan IIA improved heart function, reduced infarct size, and enhanced vascular endothelial growth factor and hypoxia-inducible factor 1alpha mRNA expression [17].

San qi, also called *Panax notoginseng*, has beneficial effects on unstable angina [18, 19]. *Panax notoginseng* saponins (PNS) are among the major lipophilic components extracted from *Panax notoginseng*. A meta-analysis and systematic review including 17 studies demonstrated that oral PNS could reduce MI, revascularization, and rehospitalization for unstable angina and improve the electrocardiography (ECG) results, frequency, and duration of angina pectoris, dosage of nitroglycerin, and lipids in unstable angina patients [19]. Multiple animal experiments have shown that PNS can improve the energy metabolism of myocardial cells and reduce myocardial damage in rats with acute MI [20–23].

Astragaloside IV (AS-IV) is the main effective ingredient of Haung-qi (Astragalus membranaceus), which has a prominent role in cardiovascular diseases. Many studies showed that AS-IV can protect against ischemic and hypoxic myocardial cell injury (by inhibiting apoptosis) [24], alleviate vascular endothelial dysfunction, and promote angiogenesis. It can also regulate blood glucose and blood lipid levels and reduce the risk of IHD [25].

The article "Chinese Herbal Medicine as an Adjunctive Therapy Improves the Survival Rate of Patients with Ischemic Heart Disease: A Nationwide Population-Based Cohort Study" was published in 2022. Journal: Evid Based Complement Alternat Med.

Da huang, also called *Rheum rhabarbarum*, is one of the most commonly used CHMs for constipation. The risk of incident IHD is higher in patients with constipation [26], and that is why Da huang is one of the most frequently used single herbs in this research.

XFZYT is a formula for promoting blood circulation. A systemic review of eight randomized controlled trials found that XFZYT combined with conventional drugs improved angina symptoms and ECG results for patients with unstable angina [27]. Experimental studies have also shown that XFZYT can increase coronary artery blood flow, improve cardiac microcirculation, prevent platelet aggregation, and accommodate blood lipids [28, 29].

ZGCT and Danshen are the most commonly prescribed CHMs for IHD in Taiwan [30]. The Cardiac Arrhythmias and Risk Stratification After Myocardial Infarction (CARISMA) trial, a multicenter observational study, found that clinically significant bradyarrhythmia and tachyarrhythmia were documented in a substantial proportion of patients with depressed left ventricular ejection fraction after acute MI. Intermittent high-degree atrioventricular block was associated with increased all-cause mortality and cardiac death [31]. The Shang Han Lun (Treatise on Febrile Diseases) notes that ZGCT activates heart-yang, restores the normal pulse, and nourishes heart-yin and blood [32]. ZGCT is widely used to treat palpitation in cases of tachycardia or bradycardia [32–34].

SMS is a well-known TCM formula used clinically to treat cardiovascular diseases [35]. It is effective for the treatment of myocardial ischemia through antioxidation, anti-inflammation, regulating Ca^2+^ homeostasis, suppressing mitochondrial mediated apoptosis, and enhancing the tolerance of ischemic tissue to hypoxia [36–38].

TWBXD and YXT have been used to treat insomnia [39–41]. Several studies have demonstrated that insomnia is associated with an increased risk of IHD, recurrent acute coronary syndrome (ACS), and mortality [42–51]. Moreover, there is a high prevalence of insomnia among patients with comorbid IHD: one-third of patients presenting with initial ACS during and after hospitalization report insomnia [47].

There were some limitations to this study. First, the NHI program contains records for only CHMs prescribed by TCM physicians, not over-the-counter CHMs, such as folk herbal remedies or decoctions. Thus, the frequency of TCM utilization may have been underestimated; we could not rule out the possibility that subjects may have taken additional herbs or agents that were not prescribed by their doctors. However, because the NHI system has comprehensive coverage of TCM prescriptions, which generally cost less than the herbs sold in Taiwan's markets, the likelihood that subjects purchased over-the-counter CHMs is low. Second, we used the ICD-9-CM codes recorded by physicians, but we had no personal history (such as smoking behavior), physical symptoms, radiological, or biochemical data to ascertain levels of disease severity. Therefore, we may have lacked data regarding important aspects that would influence the results. Third, we were unable to evaluate the safety of CHM due to the lack of data on adverse drug reactions. Although Danshen and San qi showed some interaction with anticoagulant/antiplatelet drugs in animal studies, it is still controversial in clinical use [52]. Our study revealed that these Chinese herbal medicines were still used in IHD patients frequently. There were no data to tell if the combination of CHM and anticoagulant/antiplatelet drugs would increase bleeding tendency in our study. More clinical trials are needed to verify them. Forth, we were unable to clarify the mechanism responsible for the benefits of CHM in IHD patients. Fifth, due to objections from some legislative committee members, the Health Insurance Department did not open access to information after 2010; we were unable to analyze data after 2010. Finally, though this study used propensity score matching to generate comparable CHM and non-CHM users, confounding by hypertension, hyperlipidemia, DM, stroke, or other cardiovascular diseases will be still significant concerns. For instance, specific IHD patient characteristics may preclude the use of CHM. However, the results of this study still provide valuable information; it shows that the integration of CHM and Western medicine treatments may reduce hospitalization stay and expenditure and improve survival rate.

The article "Chinese Herbal Medicine as an Adjunctive Therapy Improves the Survival Rate of Patients with Ischemic Heart Disease: A Nationwide Population-Based Cohort Study" was published in 2022. Journal: Evid Based Complement Alternat Med.

## 5. Conclusions

Combining Chinese and Western medicine treatments in IHD patients can improve 5-year survival rate, lower incurred costs, and reduce the days of hospital admission. Danshen, Huang qi, Niu xi, Da huang, and Fu zi were the most commonly prescribed Chinese single herbs; Zhi-Gan-Cao-Tang, Xue-Fu-Zhu-Yu-Tang, Tian-Wang-Bu-Xin-Dan, Sheng-Mai-San, and Yang-Xin-Tang were the five most frequently prescribed herbal formulas in Taiwan. Our findings indicate that the combination of Chinese medicine and Western medicine warrants further study.

## Figures and Tables

**Figure 1:** Flowchart of the recruitment of subjects treated with Chinese herbal medicine (CHM) from the 1 million random samples of the Longitudinal Health Insurance Database (LHID) in Taiwan.

**Figure 2:** Kaplan–Meier curve of the 10-year survival rate among Chinese herbal medicine (CHM) users and non-CHM users with ischemic heart disease (10-year survival: non-CHM users, 0.82; CHM users, 0.91).

**Figure 3:** Kaplan–Meier (a) and adjusted HR (b) landmark curves between 0 and 5 years and 5 and 12 years according to ischemic heart disease. CHM: Chinese herbal medicine.

**Table 1:** Characteristics of ischemic heart disease patients according to use or nonuse of Chinese herbal medicine.

Variable	Ischemic heart disease patients				*P* value^*∗*^
	CHM users				
	No (*n* = 20192, 50%)		Yes (*n* = 20192, 50%)		
	*n*	%	*n*	%	
CHM for IHD	—		376		
Sex					0.99
Female	8024	39.7	8024	39.7	
Male	12168	60.3	12168	60.3	

Age group					0.99
20–39	878	4.35	878	4.35	
40–64	9287	46.0	9287	46.0	
More than 65	10027	49.7	10027	49.7	
Mean ± SD (years)	63.5 (13.2)		63.4 (13.1)	0.49a	

Baseline comorbidity					
Hyperlipidemia	6275	31.1	6912	34.2	<0.001
Hypertension	12424	61.53	10496	51.98	<0.001
DM	4217	20.9	2934	14.5	<0.001
Stroke	2370	11.7	1181	5.85	<0.001

Charlson comorbidity index					<0.001
0	12921	64.0	15311	75.8	
1	3561	17.6	3238	16.0	
2	1580	7.82	881	4.36	
3+	2130	10.6	762	3.77	

Mortality	2745	13.6	1494	7.40	<0.001
Follow-up time median (IQR), years	6.00	(1.25, 6.00)	8.12	(2.77, 8.21)	<0.001^§^

IHD: ischemic heart disease; CHM: Chinese herbal medicine; DM: diabetes mellitus; SD: standard deviation. ^*∗*^Chi-square test; ^a^*t*-test. IQR: interquartile range. ^§^Wilcoxon's rank-sum test.

**Table 2:** Clinical visits for outpatient care, length of hospital stay, and medical costs for CHM and non-CHM users within 1 and 5 years after initial IHD diagnosis.

Cost	Non-CHM users		CHM users		*P* value^§^
	*n*	Mean (IQR)	*n*	Mean (IQR)	
1 year					
*Clinical visits*					
Outpatients care visits	19980	24 (15–38)	20186	29 (18–43)	<0.0001
Hospital length of stay (days)	8778	10 (4–29)	5925	6 (3–13)	<0.0001

*Cost*					
Outpatients care, NTD	19980	25708 (13150–46629)	20186	25873 (14046–44315)	0.48
Hospitalization, NTD	8778	79900 (27541–206442)	5925	41225 (20837–125302)	<0.001

5 years					
*Clinical visits*					
Outpatients care visits	20001	94 (51–150)	20191	133 (86–199)	<0.0001
Hospital length of stay (days)	13230	17 (6–52)	11648	11 (4–27)	<0.001

*Cost*					
Outpatients care (NTD)	20001	60367 (23708–128334)	20191	123496 (70499–204492)	<0.0001
Hospitalization (NTD)	13230	107436 (35341–278464)	11648	82732 (30007–212197)	<0.001

IHD: ischemic heart disease; CHM: Chinese herbal medicine; NTD: new Taiwan dollar; IQR: interquartile range.

**Table 3:** Top ten single herbs and formulas prescribed by traditional Chinese medicine physicians to treat patients with ischemic heart disease.

Herbal formula	Frequency	Number of person-days	Average daily dose (g)	Average duration for prescription (days)
*Single herb*				
Danshen	678	7730	1.4	12.2
Huang qi	264	2610	2.0	9.9
Niu xi	144	2483	1.3	17.2
Da huang	137	1435	0.4	10.5
Fu zi	137	1302	1.1	9.5
San qi	134	1061	2.3	7.9
Ji xue teng	111	2123	1.4	19.1
Hong hua	108	1734	1.2	8.4
Xu duan	107	1897	1.1	8.9
Ze xie	96	751	1.1	7.8

*CHM formula*				
Zhi-Gan-Cao-Tang	459	4861	4.5	10.6
Xue-fu-Zhu-Yu-Tang	338	3332	5.5	9.9
Tian-Wang-Bu-Xin-Dan	202	2546	4.60	12.6
Sheng-Mai-San	178	2404	4.40	13.5
Yang-Xin-Tang	137	955	8.9	7.0
Jia-Wei-Xiao-Yao-San	92	1333	3.9	14.5
Ji-Sehng-Shen-Qi-Wan	90	1511	4.70	16.8
Sheng-Mai-Yin	87	833	4.0	9.6
Zhen-Wu-Tang	84	857	8.60	10.2
Ma-Zi-Ren-Wan	75	1425	1.8	19.0

CHM: Chinese herbal medicine.

The article "Chinese Herbal Medicine as an Adjunctive Therapy Improves the Survival Rate of Patients with Ischemic Heart Disease: A Nationwide Population-Based Cohort Study" was published in 2022. Journal: Evid Based Complement Alternat Med.

**Table 4:** Hazard ratios and 95% confidence intervals of mortality risk associated with the most-used herbal products for the treatment of ischemic heart disease: a comparison of Chinese herbal medicine users and nonusers.

Prescription	*n*	Frequency of mortality	Hazard ratio (95% CI) compared with non-CHM group	
			Crude^*∗*^	Adjusted^†^
Non-CHM group	20192	2745	1 (reference)	1 (reference)
CHM group	20192	1494	0.42 (0.39, 0.45)^*∗∗∗*^	0.45 (0.42, 0.48)^*∗∗∗*^

*Single herb*				
Danshen	142	8	0.32 (0.16, 0.64)^*∗∗*^	0.28 (0.14, 0.56)^*∗∗∗*^
Huang qi	40	4	0.55 (0.21, 1.46)	0.51 (0.19, 1.36)
Niu xi	21	3	0.80 (0.26, 2.49)	0.79 (0.25, 2.45)
Da huang	18	0		
Fu zi	15	1	0.38 (0.05, 2.72)	0.33 (0.05, 2.32)
San qi	22	1	0.26 (0.04, 1.79)	0.30 (0.04, 2.14)
Ji xue teng	17	3	1.02 (0.33, 3.16)	0.83 (0.27, 2.56)
Hong hua	22	5	1.26 (0.53, 3.03)	1.05 (0.44, 2.52)
Xu duan	12	2	0.93 (0.23, 3.72)	0.83 (0.21, 3.31)
Ze xie	13	0		

*CHM formula*				
Zhi-Gan-Cao-Tang	107	9	0.51 (0.27, 0.98)^*∗*^	0.51 (0.26, 0.98)^*∗*^
Xue-fu-Zhu-Yu-Tang	95	4	0.24 (0.09, 0.63)^*∗∗*^	0.23 (0.09, 0.62)^*∗∗*^
Tian-Wang-Bu-Xin-Dan	54	3	0.31 (0.10, 0.96)^*∗*^	0.29 (0.09, 0.90)^*∗*^
Sheng-Mai-San	40	2	0.27 (0.07, 1.06)	0.26 (0.07, 1.03)
Yang-Xin-Tang	24	2	0.47 (0.12, 1.86)	0.39 (0.10, 1.56)
Jia-Wei-Xiao-Yao-San	37	2	0.31 (0.08, 1.24)	0.52 (0.13, 2.06)
Ji-Sehng-Shen-Qi-Wan	25	2	0.45 (0.11, 1.81)	0.28 (0.07, 1.13)
Sheng-Mai-Yin	33	2	0.39 (0.10, 1.57)	0.40 (0.10, 1.62)
Zhen-Wu-Tang	22	2	056 (0.14, 2.23)	0.51 (0.13, 2.03)
Ma-Zi-Ren-Wan	19	1	0.31 (0.04, 2.15)	0.25 (0.04, 1.80)

Crude HR^*∗*^ represented relative hazard ratio; adjusted HR^†^ represented adjusted hazard ratio: mutually adjusted for age, gender, hyperlipidemia, diabetes, stroke, and Charlson comorbidity index in Cox proportional hazards regression. CHM: Chinese herbal medicine; CI: confidence interval; HR: hazard ratio. ^*∗*^*P* < 0.05, ^*∗∗*^*P* < 0.01, and ^*∗∗∗*^*P* < 0.001.

The article "Chinese Herbal Medicine as an Adjunctive Therapy Improves the Survival Rate of Patients with Ischemic Heart Disease: A Nationwide Population-Based Cohort Study" was published in 2022. Journal: Evid Based Complement Alternat Med.

**Table 5:** HRs of mortality in the CHM user compared with those in the non-CHM user by Cox proportional hazard models with time-dependent exposure covariates.

CHM	Crude HR (95% CI)	Adjusted HR^†^ (95% CI)
No	1 (reference)	1 (reference)
Yes	0.07 (0.05, 0.10)^*∗∗∗*^	0.08 (0.06, 0.11)^*∗∗∗*^

CHM: Chinese herbal medicine; CI: confidence interval; HR: hazard ratio. ^*∗*^*P* < 0.05, ^*∗∗*^*P* < 0.01, and ^*∗∗∗*^*P* < 0.001.

**Table 6:** Incidence rates, hazard ratio, and confidence intervals of mortality for with and without CHM used anomaly patients in the stratification by gender, age, baseline comorbidity, and Charlson comorbidity index.

Variables	Ischemic heart disease patients						Crude HR	Adjusted HR
	Non-CHM user (*N* = 20192)			CHM user (*N* = 20192)				
	Event	Person-years	IR^†^	Event	Person-years	IR^†^	(95% CI)	(95% CI)^‡^
Sex								
Female	983	51471	19.1	513	66613	7.70	0.40 (0.36, 0.44)^*∗∗∗*^	0.46 (0.41, 0.51)^*∗∗∗*^
Male	1762	77352	22.8	981	98565	9.95	0.43 (0.40, 0.47)^*∗∗∗*^	0.45 (0.41, 0.48)^*∗∗∗*^

Age								
18–39	31	6460	4.80	11	7248	1.52	0.32 (0.16, 0.63)^*∗∗*^	0.41 (0.21, 0.83)^*∗*^
40–64	634	66699	9.51	191	76927	2.48	0.26 (0.22, 0.31)^*∗∗∗*^	0.32 (0.27, 0.37)^*∗∗∗*^
More than 65	2080	55665	37.4	1292	81004	16.0	0.42 (0.39, 0.45)^*∗∗∗*^	0.48 (0.45, 0.51)^*∗∗∗*^

Baseline comorbidity								
No	1568	1077048	14.7	1145	144550	7.92	0.53 (0.49, 0.57)^*∗∗∗*^	0.47 (0.43, 0.51)^*∗∗∗*^
Yes	1177	21776	54.1	349	20629	16.9	0.32 (0.28, 0.36)^*∗∗∗*^	0.31 (0.27, 0.34)^*∗∗∗*^

Charlson comorbidity index								
0	994	93509	10.6	848	128473	6.60	0.60 (0.55, 0.66)^*∗∗∗*^	0.54 (0.49, 0.59)^*∗∗∗*^
1	686	20412	33.6	380	25505	14.9	0.43 (0.38, 0.48)^*∗∗∗*^	0.41 (0.36, 0.47)^*∗∗∗*^
2	410	7245	56.6	133	6323	21.0	0.37 (0.30, 0.45)^*∗∗∗*^	0.37 (0.30, 0.45)^*∗∗∗*^
3+	655	7657	85.5	133	4877	27.3	0.33 (0.28, 0.40)^*∗∗∗*^	0.32 (0.26, 0.38)^*∗∗∗*^

IR, incidence rates, per 1,000 person-years; HR, hazard ratio; CI, confidence interval ^†^adjusted for CHM used, age, gender, baseline comorbidity, and Charlson comorbidity index in Cox proportional hazards regression ^*∗*^*P* < 0.05; ^*∗∗*^*P* < 0.01; ^*∗∗∗*^*P* < 0.001.

## Data Availability

No data were used to support the findings of the study.
